# A Fast CS-Based Reconstruction Model with Total Variation Constraint for MRI Enhancement in K-Space Domain

**DOI:** 10.1155/2022/9222958

**Published:** 2022-07-06

**Authors:** Hongxuan Duan, Xiaochang Lv

**Affiliations:** ^1^Northeast Petroleum University, Daqing 163318, China; ^2^Northeast Petroleum University of Qinhuangdao, Qinhuangdao 066004, China

## Abstract

Due to the fact that Magnetic Resonance Imaging (MRI) is still a relatively slow imaging modality, its application for dynamic imaging is restricted. The total variation is introduced into the CS-based MRI reconstruction model, and three regularization conditions are adopted to ensure that a high-quality reconstructed image is produced. In this paper, a simple yet fast CS-based optimization model for noisy MRI Enhancement is proposed. The alternative direction multiplier method is chosen to optimize the model, and the *k*-terms power series is applied in order to derive the LogDet function into the augmented Lagrange form. Following this, an approximation of the feature vector is achieved through the iterative process. The quality of the reconstructed image was much better than that of the CS-based MRI image reconstruction algorithm, as shown by experimental results under different noise conditions. The peak signal-to-noise ratio of the reconstructed image was able to be improved anywhere from 5 to 20 percent.

## 1. Introduction

Since the excited hydrogen nucleus will release its energy by emitting a signal with a specific frequency, the signal can be detected and reconstructed by corresponding MRI technical so as to recover the internal image data, which makes it possible for the rapid examination and reasonable diagnosis of diseases [1]. However, MRI will invariably have issues with noise, and the reduction in the number of phase-encoded signals will result in truncation artifacts when the truncated K-space data is Fourier transformed to reconstruct the image. This will have a direct impact on how accurately the image is analyzed, as well as the results of any subsequent medical diagnosis. It is of the utmost importance to determine how to process the noisy MRI enhancement in a reasonable and accurate manner [2].

The essence of MRI enhancement is that the detailed information of the image is fully reserved, and the irrelevant information such as noise and artifacts is removed to the greatest extent. At present, most MR image enhancement methods assume that the interference signal obeys Gaussian distribution and many effective enhancement algorithms are proposed. The enhancement algorithms for MRI images can, as of right now, be broken down into three distinct categories. The first type is known as the variational-based method, and it is distinguished by the fact that it realizes MRI enhancement by finding the numerical solution to a particular partial differential equation. Some examples of this type of method include the adaptive anisotropic diffusion enhancement method, the fractional total variation enhancement model with L1 fidelity, and the minimum unbiased risk estimation for MRI enhancement. In order to find a solution to the issue of MR image enhancement, Chen et al. utilized the total variation regularization (TV) model. The ability of total variation mode of effectively eliminating random noise while simultaneously preserving the image's edges is the primary benefit of utilizing this mode [3–5]. On the other hand, in order to use the total-variation method, MR images need to fulfill the requirements of piecewise constancy. This requirement cannot be satisfied in the actual MRI system because there is a nonuniformity between the high field system and the excitation B1 field of 3T. In addition, the enhancement method that is based on total variation will, under the assumption of piecewise invariance, result in the emergence of an artificial effect, which will cause the reconstruction result to be artificial. This is because the assumption states that piecewise invariance exists. The name of the second approach is the transform domain method. Its most distinguishing characteristic is the ability of eliminating interference in the transform domain and then performing an inverse transform in order to obtain an image of superior quality using techniques such as the wavelet threshold transformation method, different shrinkage criteria methods of wavelet transform, and the wavelet transform approach for MRI enhancement. According to the research in [6], the MR image can be improved and denoised through the use of bilateral filtering in the wavelet domain. However, the improved result will show pseudo-Gibbs phenomenon at the point where the signal discontinues. The third one is referred to as the NLM enhancement method, and it is typically distinguished by the application of a significant quantity of spatially redundant information. Initially, the NLM algorithm was utilized primarily for the purpose of addressing Gaussian distributed noise. It is able to reserve more details and remove more noise than general methods because it has obvious advantages over those methods. In recent years, NLM and its improved algorithm have been applied to MR images and have achieved a good enhancement effect. Some examples of this include nonlocal enhancement based on the Gaussian model, maximum likelihood nonlocal estimation method, and nonlocal enhancement based on unbiased estimation [7, 8].

Although high-quality MRI images can be obtained by enhancement algorithms, most of these algorithms still analyze and process the images and do not make use of the essential features of MRI raw data. It is well known that the generation of MRI requires three main steps: (1) the protons in the imaging area generate signals (FID signal, SE signal, STE signal, etc.) through the cooperation of RF pulse and gradient magnetic field; (2) the MRT/R coil is adopted to acquire these signals and fill the acquired signals into the K-space; (3) Fourier transform is performed on the data in K-space to obtain a magnetic resonance image. Therefore, the K-space is the space for storing the original data of magnetic resonance, and the magnetic resonance image can be obtained by performing very complex data postprocessing on the original data of the K-space. Therefore, some scholars began to explore the data processing in K-space so as to improve the signal quality in the imaging process [9].

In an MRI system, image signals are recorded sequentially in K-space. The scanning efficiency is the most important factor in determining how quickly images can be acquired in this system. Because of the MRI system's slow data acquisition speed, motion artifacts and noise are both relatively simple to generate. According to CS theory, if a signal is compressible or sparse in a transform domain, the high-dimensional signal can be mapped into the low-dimensional space using an observation matrix unrelated to the transform basis, and the original signal can be reconstructed with a high probability from a small number of projections by solving the optimization problem. This is done by mapping the high-dimensional signal into low-dimensional space. The application of CS theory should make it possible to drastically cut down on the amount of data acquired, significantly cut down on the amount of time spent acquiring data, and guarantee high-quality image reconstruction. Lustig et al. applied CS theory to MRI for the first time, where the undersampled MR image reconstruction is expressed as a *l*_0_ norm minimization problem, and solved it by greedy algorithm. The *l*_0_ norm minimization problem is a NP hard problem. Lustig relaxes the *l*_0_ norm problem to the *l*_1_ norm problem and uses the conjugate gradient method to solve it. In order to improve the speed and accuracy of image reconstruction, it applies total variation to CS-based MRI model and uses two regularization conditions to ensure high-quality reconstructed image. Wang et al.introduce the dual-tree complex wavelet to obtain the global sparsity priori, combined with CS theory to reconstruct the MR image with directional structure, but the comprehensive sparse coding phase in its solution process takes a long time, resulting in the low efficiency of MRI enhancement reconstruction. With the advent of compressed sensing (CS) theory, minimizing the recording time in K-space without affecting the image quality has become the main purpose for MRI enhancement research. Due to the effective use of signal sparsity, the K-space samples required for MR image reconstruction are far less than those of conventional methods. Furthermore, it can significantly reduce the scanning time, making it a popular fast imaging method. Nowadays, compressed sensing theory has been successfully applied to MRI reconstruction [10]. In CS-based MRI enhancement algorithm, the adaptive sparse representation of MR image plays an important role in high-quality image reconstruction. The adaptive sparse representation of MR image refers to learning by using the training samples of known MR image, so as to obtain the adaptive dictionary matching with MR image. The adaptive sparse representation of MR image can obtain accurate sparse priors and capture rich structural information of the image. In recent years, MRI enhancement algorithm based on adaptive sparse representation model has become the research direction. These improved CS-based algorithms can reconstruct MR images more accurately, but these algorithms have some defects, which still need to be further improved. As a result, with the assistance of computer science theory, the purpose of this paper is to conduct an in-depth investigation of the adaptive sparse representation model in order to increase the speed of image reconstruction while simultaneously enhancing its overall quality.

In this paper, a straightforward and speedy CS-based optimization model for noisy MRI Enhancement is proposed. In this model, the total variation is incorporated into the CS-based MRI reconstruction model, and three regularization conditions are utilized to ensure that the reconstructed image is of high quality. In order to quickly solve the objective function, the alternative direction multiplier method is utilized to optimize the model. Additionally, the *k*-terms power series is implemented in order to derive the LogDet function into the augmented Lagrange form, and finally an approximation of the feature vector is achieved through the iterative procedure.

## 2. Radial Subsampling and Its K-Space in MRI System

As we all know, accelerating the speed of imaging has always been the focus of Magnetic Resonance Imaging research, which can not only improve the efficiency of MRI system, but also weaken or eliminate motion artifacts and noise, so that MRI can be better applied to medical diagnosis [6, 11–13]. In MRI system, there are generally two methods to shorten the time of data acquisition: one is to use multichannel parallel imaging technology; the other is to use non-Cartesian sampling trajectory to fill K-space, such as radial subsampling and sparse sampling [14–17].

Radial subsampling in MRI data acquisition is to collect magnetic resonance data in a radial trajectory rather than parallel linear manner. Radial subsampling not only changes the phase coding gradient and adopts sinusoidal gradient magnetic field, but also uses two coding gradient magnetic fields, *G*_*x*_ and *G*_*y*_, so that the direction of the total gradient vector forms an arbitrary angle *θ* with the *x*-axis. Therefore, the total gradient intensities *G* and *θ* in the two directions are

(1) $$\begin{array}{c} G=\sqrt{G_{x}^{2}+G_{y}^{2}},\\ \theta =\text{arctan}\left(\frac{G_{y}}{G_{x}}\right). \end{array}$$

Radial subsampling should also meet Nyquist sampling theorem. The difference of sampling steps will lead to the existence of aliasing artifacts in image reconstruction. In radial subsampling, the first two parameters *G* and *θ* cannot be directly converted into spatial resolution. Since the former depends on the number of radial lines *n*_*s*_, the parameters can be set freely in actual sampling. Generally, the number of radial lines is set to *n*_*s*_, so it can be denoted by

(2) $$\begin{array}{c} n_{s}=\frac{\pi n}{2}. \end{array}$$

Satisfy the above formula to ensure that the maximum distance between adjacent radial subsampling lines is not greater than Δ*k*. Since traditional MRI uses Cartesian trajectory, its reconstruction method is simple, but line by line acquisition is very sensitive to motion artifacts. Non-Cartesian sampling, such as radial sampling, has obvious advantages over Cartesian sampling. There are mainly the following two aspects: firstly, each line of radial sampling data contains the same amount of low-frequency to high-frequency information, which is conducive to the subsampling reconstruction of MRI images. Secondly, the radial sampling mode determines its oversampling of K-space center data, and K-space center data determines the main information of the image. Therefore, radial sampling is not as sensitive to the motion parameter. However, radial sampling also has some disadvantages. For example, the radial sampling trajectory is densely sampled in the middle and sparsely sampled at the edge, and then the sampling density is uneven. Therefore, the image cannot be obtained directly by Fourier transform, so the imaging process is more complex. It is necessary to use grid interpolation method or Zero_filling strategy to interpolate the data to uniform grid points and then perform Fourier transform to obtain the final image. Radial subsampling and its MRI image are shown in Figure 1. The specific operation can be seen in [18].

K-space is the space for storing the raw data of magnetic resonance, and the magnetic resonance image can be obtained by performing very complex data postprocessing, as shown in Figure 1. After the radial sampling data set is interpolated into the Cartesian coordinate system by gridding convolution, the resampled data can be directly used to obtain the final MRI reconstruction image by inverse fast Fourier transform. It can be seen that there is no one-to-one corresponding relation between the array points in the K-space and the reconstructed pixel points in image space. But the frequency encoding direction and phase encoding direction of K-space are symmetrical. Due to the spatial positioning effect of the gradient field in the phase encoding direction, the phase encoding gradient in the center of K-space is zero, and the phase encoding on both sides increases in turn, so it is also symmetrical in *t*. This is because in the frequency encoding direction a continuous curve that is composed of many signal subsampling points is collected, and the curve is a symmetrical curve, so it is symmetrical in the frequency encoding direction. Each point in the K-space corresponds to all of the pixels in the MR image, and the image contrast is determined by the central part of the K-space, while the spatial resolution is determined by the peripheral part of the K-space. Theoretically, one can obtain a quarter of a subsample of the K-space, and then the remaining space can be filled mathematically, which results in an MRI image. This can result in phase errors and image distortions as a result of errors and noise in the data acquisition process. The challenge that needs to be tackled is figuring out how to carry out image reconstruction and enhancement with only a limited amount of data in order to obtain MRI data of a high quality. The CS-based MRI enhancement model is improved with the help of a powerful and efficient optimization algorithm that is used in this paper.

## 3. K-Space Enhancement Reconstruction Algorithm for Noisy MRI

### 3.1. Improved CS-Based MRI Model

In an MRI system, image signals are recorded sequentially in K-space. The scanning efficiency is the most important factor in determining how quickly images can be acquired in this system [19]. Because of the MRI system's slow data acquisition speed, motion artifacts and noise are both relatively simple to generate. According to the CS theory, if the signal in a transform domain is compressible or sparse, the high-dimensional signal can be mapped into the low-dimensional space using an observation matrix that is unrelated to the transform basis, and the original signal can then be reconstructed with a high probability from a limited number of projections by solving the optimization problem. By mapping the high-dimensional signal into the low-dimensional space, this is achieved. In the theory of CS, the image reconstruction model can be expressed as *Y*=Φ*X*, where *X* is an image matrix; Φ ∈ *R*^*M*×*N*^ is an observation matrix; *Y* is a measurement matrix. When *M* < *N*, this means that many solutions can be obtained for the equation *Y*=Φ*X*. In order to constrain the results, it is generally necessary to add regularization terms to the equation, such as total variation, sparse, and BM3D.

If the image is sparse under the representation of a dictionary, and its model can be written as *X*=*DA*, where *A* is a sparse matrix and *D* is a dictionary, it can be solved by using an appropriate sparse optimization algorithm, and then the image *X* can be reconstructed by solving the *X*=*DA*. In the image inverse problem based on CS construction, selecting an appropriate dictionary plays a key role in image reconstruction.

MRI images are sparse in a specific transform domain, which meets the requirements of CS theory for signal sparsity. The convex optimization problem of l1 norm is constructed in combination with compressed sensing theory. It can be concluded that the objective function of CS-based MRI reconstruction is

(3) $$\begin{array}{c} \hat{x}=\underset{x}{\text{argmin}}\frac{1}{2}\left\|Fx-y\right\|+\lambda \text{L}\left(x\right), \end{array}$$

where *x* is the MRI image to be reconstructed, *F* represents the Fourier transform operator, and *y* is the K-space data obtained after MRI scanning; *L*(*x*) is the regularization term. According to the distribution of the signals in the K-space data, the corresponding sparse transform domain, the observation matrix and the appropriate CS-based reconstruction algorithm are selected. The MRI image can be reconstructed by solving the CS-based enhancement algorithm for (3). However, to improve the reconstruction accuracy, many effective objective functions have been proposed, such as sparse and low-rank regularization constraints. The nonlocal group-sparse model proposed by Dong et al. is the most famous [2], whose global objective function is shown as follows:

(4) $$\begin{array}{c} \left(\hat{x},L_{i}\right)=\underset{x,L_{i}}{\text{argmin}}{\left\|\Phi x-y\right\|}_{2}^{2}+\eta \sum_{i}\left({\left\|R_{i}x-L_{i}\right\|}_{2}^{2}+\lambda \text{L}\left(x\right)\right), \end{array}$$

where *R*_*i*_*x*_*i*_ is expressed as a low-rank matrix composed of all nonlocal similar patches of the sample *x*_*i*_. In order to solve the multivariable objective function, the idea of alternating solution is adopted to optimize, which fixes one variable to solve another variable and finally obtains the optimal solution. Although the objective function in (4) can achieve better performance than the traditional CS-based enhancement, it can only be effective for Gaussian distribution, and the solution process is extremely complex. TV regularization model is one of the most successful image reconstruction models, which can adapt the noisy data with different distribution for reconstruction and enhancement. In order to adapt to different noise distributions and accelerate the solution speed, the improved objective function proposed in this paper is as follows.

(5) $$\begin{array}{c} \left(\hat{x},L_{i}\right)=\underset{x,L_{i}}{\text{argmin}}{\left\|\Phi x-y\right\|}_{2}^{2}+\eta \sum_{i}\left({\left\|R_{i}x-L_{i}\right\|}_{2}^{2}+\lambda \text{L}\left(x\right)\right)+\beta \int_{\Omega }\left|\Phi x-y\right|\text{d}x. \end{array}$$

It can be seen that the improved model in this paper introduces the total variational regularization on the basis of (5). However, it is not easy to solve, so we relax the constraints; *i.e.,*∫_Ω_|Φ*x* − *y*|d*x*=〈Φ*x* − *y*, z〉. As a consequence, we can adopt the alternative direction multiplier method for solving (6).

Firstly, split (6) and rewrite it into the augmented Lagrange form.

(6) $$\begin{array}{c} \left(\hat{x},L_{i}\right)=\underset{x,L_{i}}{\arg\min}{\left\|\Phi x-y\right\|}_{2}^{2}+\eta \sum_{i}\left({\left\|R_{i}x-L_{i}\right\|}_{2}^{2}+\lambda L\left(x\right)\right)+\beta \langle \Phi x-y,z\rangle , \end{array}$$

where *z* is Lagrange multiplier; *γ*, *η*, *β* are penalty factors. (*x*^*k*^.*x*^*k*^, *z*^*k*^) is iterated through the alternative direction multiplier method and get (*x*^*k*+1^.*y*^*k*+1^, *z*^*k*+1^)，whose step is shown as follows:

(7) $$\begin{array}{c} \left\{\begin{array}{c} \left(x^{k+1},y^{k+1}\right)\leftarrow \underset{x\in R^{n},y\in rR^{n}}{\text{argmin}}L_{\gamma }\left(x.y.z^{k}.\gamma \right),\\ z^{k-1}\leftarrow z^{k}-\gamma \left(x^{k-1}-y^{k-1}\right). \end{array}\right) \end{array}$$

It is worth noting that (7) only regards ((6) as a general linear constrained convex programming problem without considering its separable structure, so it is necessary to solve two variables *x*^*k*+1^ and *y*^*k*+1^ at the same time. On the contrary, the alternative direction multiplier method decomposes (7) into two subproblems to solve *x*^*k*+1^ and *y*^*k*+1^, respectively, so it has the following form:

(8) $$\begin{array}{c} \left\{\begin{array}{c} y^{k+1}\leftarrow \text{argmin}L_{\gamma }\left(x.y^{k}.z^{k}\right),\\ x^{k+1}\leftarrow \text{argmin}L_{\gamma }\left(x^{k+1}.y.z^{k}\right),\\ z^{k+1}\leftarrow z^{k}-\gamma \left(x^{k+1}-y^{k+1}\right). \end{array}\right) \end{array}$$

In other words, the subproblem for solving *x* can be rewritten as

(9) $$\begin{array}{c} x^{k+1}=\underset{x\in R^{n}}{\text{argmin}}\left\{\frac{1}{2}{\left\|\Phi x-y\right\|}^{2}+\left\|x-y^{k+1}-\frac{z^{k}}{\gamma }\right\|\right\}. \end{array}$$

Therefore, in order to solve the MRI enhancement problem under the background of least squares problem by using linear alternative direction multiplier method, (*τ*/2)‖*x* − *x*^*k*^‖^2^ is introduced into the subproblem, so *x*−subproblem can be solved by computing

(10) $$\begin{array}{c} x^{k+1}=\arg\underset{x\in R^{n}}{\min}\left\{\frac{1}{2}{\left\|\Phi x-y\right\|}^{2}+{\left\|x-y^{k+1}-\frac{z^{k}}{\gamma }\right\|}^{2}+\frac{\tau }{2}{\left\|x-x^{k}\right\|}^{2}\right\}, \end{array}$$

where *τ* > *ρ*(Φ^*T*^Φ) is positive constant. Therefore, the weighted singular value thresholding operator can be adopted to solve optimization result, as in [2].

In this paper, the total variational constraint is introduced into nonlocal group-sparse model, and the parameters of the objective function are relaxed, so that each subproblem can have analytical solutions, and the size of iterative step is greater than 1. For example, *z*^*k*+1^ has a closed-form solution; we can obtain

(11) $$\begin{array}{c} \left\{\begin{array}{c} y^{k+1}\leftarrow \frac{1}{\lambda^{2}\Phi^{T}\Phi +\gamma I}\left(\lambda^{2}\Phi^{T}y-z^{k}+\gamma x^{k}\right),\\ x^{k+1}\leftarrow P_{\Omega }\left\{\frac{1}{\tau +\gamma }\left[\tau x^{k}+z^{k}+\gamma \left[\omega y^{k+1}+\left(1-\omega \right)x^{k}\right]-A^{T}\left(Ax^{k}-b\right)\right]\right\},\\ z^{k+1}=z^{k}-\gamma \left[x^{k+1}-\omega y^{k+1}-\left(1-\omega \right)x^{k}\right], \end{array}\right) \end{array}$$

where *ω* ∈ (0,2) is the relaxation operator.

### 3.2. LogDet Optimization for Acceleration

To solve the improper operation of hard threshold for all singular values, the smoothing effect caused by inaccurate estimation of matrix rank, and the high time complexity of the algorithm caused by a large number of iterative optimizations, we use the LogDet optimization for acceleration to estimate the singular value, so we can directly obtain the singular value approximation based on the number of singular value iterations.

In [6], it has been proved that low-rank problem can be approximated to LogDet problem. For a general matrix *L* that is neither square nor positive semidefinite, it can be slightly modified as *L*(*X*)=logdet((*XX*^T^)^1/2^+*εI*). Because of *XX*^T^=*U*Σ*U*^T^, so we can obtain *L*(*X*)=logdet(Σ^1/2^+*εI*), where Σ is diagonal matrix composed of singular values of *XX*^T^. In other words, we can use the LogDet optimization to replace low-rank model, which can improve optimization speed. However, when the matrix decomposition method is used for *XX*^T^, its computation complexity of the exact solution is 0(*N*^3^), so its computational cost and additional storage requirements may limit their use in MRI real-time reconstruction.

Literature [20] proposed a uniform distributed sample selection method for the estimation of random traces in the process of Gaussian regression, whose computation complexity of the exact solution for logdet function is just a O(*N*^2^). In the decomposition of large sparse matrix, logdet(C) can realize the approximation estimation based on power series expansion. Since any matrix can be converted into a specific form *I* − *a*  *D*, its eigenvalues remain less than 1 after row standardization or extraction of a sufficiently large factor, where, *a* ∈ (0,1), *I* and *D* are expressed as identity matrix and large sparse matrix, respectively. Firstly, the power series expansion method is applied to the approximation of generalized positive definite matrix, and then the power series truncation error compensation is used, and its result can be used as an effective surrogate function for accurate estimation. For a positive definite matrix *C* ∈ *R*^*N*×*N*^, the approximate value of the *k*-terms power series for logdet(*C*) can be denoted by

(12) $$\begin{array}{c} \text{logdet}C\approx N\text{log}\left(a\right)-N\varepsilon \left(\sum_{i=1}^{k}\frac{s^{T}B^{i}s}{is^{T}s}\right), \end{array}$$

where *a*=‖*C*‖_*∞*_, *B*=*I* − *C*/*a*, *s* ~ *N*_*N*_(0, *I*).

On basis of the infinite norm of the matrix, we can obtain

(13) $$\begin{array}{c} \text{logdet}\left(C\right)=\text{logdet}\left(aA\right)=\text{log}\left(a^{N}\text{det }A\right)=N\text{ log}\left(a\right)+\text{logdet }A, \end{array}$$

where *α*=‖*C*‖_*∞*_=max_*i*_(∑_*j*=*i*_^*N*^*c*_*ij*_), and *A*=*C*/*a*. Therefore, logdet *A* can be approximately expressed as the sum of a simple polynomial

(14) $$\begin{array}{c} \text{logdet }A\approx -N\varepsilon \left(\sum_{i=1}^{k}\frac{s^{T}B^{i}s}{is^{T}s}\right), \end{array}$$

where *ε* is the mean for random number. The basic algorithm of logdet(*C*) is based on equations (13) and (14), where an intermediate vector *ν* needs to be calculated or stored; that is, *ν*^*t*+1^=*Bν*^*t*^ and *ν*^0^=*s*. The above approximate estimation method only needs O(*N*^2^) operations and *N* vector storage. Compared with the traditional matrix decomposition, our adopted strategy can meet the needs of MRI data reconstruction in K-space.

## 4. Experiments

### 4.1. Parameter Setting

In order to verify the effectiveness of the proposed noisy MRI reconstruction algorithm in K-space, this section report the experimental results for simulation comparison experiment. In this experiment, six MRI images are selected for testing, and the noise variance is 5, 10, 25, and 50 respectively. In the experimental parameters, the size *f* of image patch and the size *W* of search window are *σ*^2^ < 30*f*  = 7， *W*  = 21; *σ*^2^ ≥ 30， *f*  = 9， *W*  = 31. Since the number of similar patches is adaptive, it overcomes the introduction of dissimilar image blocks due to the fixed number of similar patches, but too many similar blocks will increase the amount of calculation, so we set the boundary value *S*_*i*_ ∈ [10,60]. The regularization parameter *λ*, *β*, *η* is tuned separately for different iteration times, where the initial values are set to 0.1, 0.05, and 0.01, respectively. Sensing rate in K-space is set to 0.05, 0.1, 0.2, 0.3, 0.4, 0.5, and 0.6. Noisy MRI reconstruction algorithms are programmed using MATLAB language. The experimental simulation platform is a personal computer with Intel (R) core (TM) i5 dual core CPU, 2.6 GHz frequency, 4G memory, Win10 operating system and MATLAB 2017a is selected as experimental simulation software.

### 4.2. Evaluation Indexes

Some common objective evaluation indexes for performance quantification have been adopted in order to perform an objective evaluation of the reconstruction performance of the improved reconstruction algorithm for noisy MRI with different noise distributions. These objective evaluation indexes include mean square error (MSE), peak signal-to-noise ratio (PSNR), and structure similarity (SSIM). Since MSE is the divergence of the mean square error between the original picture and the reconstructed image, its primary application is in the simulation experiment of a known original image.

(15) $$\begin{array}{c} MSE=\sum_{i\in I}{\left|x\left(i\right)-\hat{x}\left(i\right)\right|}_{2}^{2}, \end{array}$$

where $\hat{x}$ represents the reconstructed gray level. MSE reflects the approximation degree of the reconstructed image to the original image. The smaller its value is, the better the noisy MRI construction effect is.

Peak signal-to-noise ratio is an image-quality evaluation index based on mean square error, which is defined as

(16) $$\begin{array}{c} PSNR=10\mathrm{lg}\left[\frac{255^{2}}{\sum_{i\in I}{\left(x\left(i\right)-\hat{x}\left(i\right)\right)}^{2}/\text{M}\times N}\right], \end{array}$$

where *M*, *N* represent the size of image. It can be seen from the (15) and (16) that the evaluation of PSNR and MSE is just the opposite. The larger PSNR the better reconstruction result, and the smaller PSNR the worse reconstruction effect.

Structural similarity is to evaluate the performance of image reconstruction algorithm from the perspective of the edge structure of image, which evaluates the quality of image based on structural distortion. It is an objective evaluation method very close to human vision, which is defined as follows:

(17) $$\begin{array}{c} \text{SSIM}=\frac{4u_{x}u_{y}\sigma_{xy}}{\left(u_{x}^{2}+u_{y}^{2}\right)\left(\sigma_{x}^{2}+\sigma_{y}^{2}\right)}, \end{array}$$

where *u*_*x*_, *u*_*y*_ represent the mean value of the original image and reconstructed image, respectively; *σ*_*x*_, *σ*_*y*_ can represent the variance of the original image and the estimated image, respectively. If the two structures are more similar, the value of SSIM is greater, and the value of SSIM is less than or equal to 1.

### 4.3. Reconstruction Performance for Different Noises

To verify the performance of the improved algorithm for noisy MRI reconstruction with different noise distributions, Rayleigh noise, Gaussian white noise, and random nonuniform noise are selected for reconstruction analysis, where the standard deviation *σ*_*n*_ of Gaussian noise is 5, 15, 25, 20, and 35, respectively. All of the comparison tests had their noisy images treated using the same settings. We also performed a comparison study of the experimental outcomes, looking at them from both a subjective and an objective perspective. During the subjective evaluation, the smooth area and the area with rich texture information are primarily selected for analysis, and the performance of the reconstruction method is evaluated based on the visual effect. During the objective evaluation, PSNR and SSIM are utilized in order to evaluate the performance of the reconstruction effect.

Uniform noise is defined as noise that obeys the same distribution at different pixel positions of the image; namely, the distribution of any position (*i*, *j*) is the same in *y*=*x*+*n*. Nonuniform noise is defined as the noise that either obeys different distributions at different pixel positions or obeys the same distribution but has different corresponding parameters. The noise *n*_*ij*_=*nδ*_*ij*_ at any position (*i*, *j*) in the image *y*=*x*+*n* obeys different distributions or has the same distribution but different parameters, where the value of the sampling function *n*_*ij*_=*nδ*_*ij*_ at any position (*i*, *j*) is 1 and 0 at other positions. For the convenience of discussion, the standard deviation *σ* of nonuniform Gaussian noise follows the uniform distribution of [1 : 100], while the standard deviation of uniform Gaussian noise is *σ*=20.  Table 1 shows the reconstruction results under different noise distributions. NL-CS and GSCS are the selected comparison algorithms, where NL-CS is a reconstruction algorithm based on nonlocal compressed sensing and GSCS is a group-sparsity based reconstruction algorithm. The best results in Table 1 have been bold. It can be seen that the reconstruction performance of the reconstruction algorithm proposed in this paper is the best under different types of noise, because the regularization constraints used in this paper are independent of the noise model, while the comparison models are optimized based on Gaussian noise model. The processing ability of NL-CS and GSCS for Gaussian noise is significantly better than that of the other two kinds of noise in Table 1.

It is evident from the results of the reconstruction shown in Figure 2 that our approach does a better job of preserving the features. When compared to NL-CS, it is only slightly poorer in the bright places, but when compared to other comparative algorithms it performs significantly better in the bright spots. The noise in the image is exceedingly chaotic as a result of the interference caused by the nonuniform Gaussian noise. The noise can be effectively separated using the model that was proposed in this study. The reconstruction performance is capable of preserving the detailed signal, particularly in the edge region, but there are also fake effects in some locations. This is especially true for the edge region. Some of the highlighted noise spots in the amplification region are smoothed down in the salt and pepper noise area; however the comparison process has a lot of interference, and the reconstruction impact is not very good.  Figure 3 is the comparison of reconstruction residual for Gaussian noise with *σ*=20, where the proposed model has the least texture detail and the best reconstruction performance.

### 4.4. Comparison of Reconstruction Performance for Different Algorithms

To verify the performance of noisy MRI enhancement reconstruction in K-space, we selected some representative comparison algorithms, such as KLLD, SAIST, LSSC, NL-CS, and GSCS. The low-rank algorithms of KLLD reconstruction in solving RPCA model are singular value threshold operations based on hard threshold, and the low-rank matrix is obtained through repeated iterations. Our method is mainly to solve the improper operation of hard threshold for all singular values, the smoothing effect caused by inaccurate estimation of matrix rank, and the high time complexity of the algorithm caused by a large number of iterative optimizations. We use the LogDet optimization for acceleration to estimate the singular value, so we can directly obtain the singular value approximation based on the number of singular value iterations. SAIST is to solve the problem that LSSC needs to establish a very large redundant dictionary, resulting in too high spatial complexity and too high time complexity by solving it through low-rank algorithm on the basis of dictionary. Since the signal space can be divided into noise-free signal space and noise space, and the peak of the singular value difference curve is the critical point of the signal space, we used the LogDet optimization to divide the similarity matrix into low-rank part and difference part. The singular values corresponding to the low-rank part account for the vast majority of the sum of all singular values, and the proportion of noise pollution is small. Based on the prior information, we use the *k*-terms power series to split and rewrite the LogDet function into the augmented Lagrange form and then approximate the real vector in the iterative process. Finally, it can be seen that the improved CS-based MRI reconstruction algorithm can approximate the real noise-free data.  Table 2 shows that, compared with NL-CS, KLLD, and GSCS, our algorithm can effectively reduce noise, improve denoising performance, and save texture edge and other structural information. When the noise is less than 15, our algorithm PSNR is much higher than NL-CS, KLLD, and GSCS about 0.2 dB. With the increase of noise intensity, the advantage of our algorithm weakens, but it is also equivalent to the best algorithm, which is due to the preservation of texture and the smoothing effect of smooth area. However, since our algorithm is based on LogDet optimization for acceleration, the reconstruction time of the algorithm is the best.

For the irregular texture image, such as head MRI, our algorithm can retain the texture structure but ignore the small details. Even so, our algorithm is better than the comparison algorithm. NL-CS algorithm is not denoised enough in the texture area. Although the texture information is still saved, the reconstruction result is incomplete. Although the evaluation index of NL-CS and GSCS is greatly improved compared with KLLD, both methods are based on the sparse coefficients under the CS dictionary. Due to the pseudo-Gibbs effect, there are more scratches in the smooth area. Our method mainly deals with LogDet function, and Gibbs effect is inevitable, but we adjust the threshold according to the mode characteristics of the image patch to further improve our reconstruction quality; especially the TV model is introduced to separate the residual matrix of the similar patches. Our proposed algorithm performs much better than the comparison algorithms on all noisy images and sensing rates.

### 4.5. Ablation Analysis

The comparison of the PSNR of the reconstructed picture using the proposed technique for various sensing rates of an MRI image is shown in Figure 4. The ordinate represents the number of iterations, and there are a total of one hundred iterative tests performed.  Figure 5 demonstrates that the quality of the reconstructed picture for 0.4 sensing rate and 0.5 sensing rate is comparable to one another; however the quality of the reconstructed image for 0.6 sensing rate is noticeably superior to that of the other two sensing rates. A sensing rate of 0.6 is chosen for the radial subsampling lines because the goal of the ablation analysis is to lower the sensing rate in order to enhance the reconstruction quality and efficiency under the conditions without compromising the performance of the hardware.

In addition to the number of iterations, take the size parameter of overlapping patches as an example. We also analyze the results of reconstruction experiments under three different overlapping patch sizes 6 × 6, 7 × 7, and 8 × 8. It can be seen that the PSNR of reconstructed images corresponding to the three patch sizes is not much different, but the SSIM of 8 × 8 is the best, and the growth range of PSNR is decreasing. Considering the calculation cost, 8 × 8 is selected as the size of overlapping patches. By experiment contrast, our proposed algorithm can preserve the edges and local structures better than comparison algorithms. This paper adopts LogDet optimization for acceleration. In order to analyze the reconstruction efficiency, the algorithm using low-rank decomposition is recorded as LR-CS, and the nonconvex LogDet surrogate of the rank is recorded as Logdet_CS. In order to facilitate ablation analysis, the algorithm model is consistent except that different methods are used to solve the low-rank module. We also analyze the reconstructed PSNR and reconstruction time under different iterations. It can be seen that the PSNR of different comparison algorithms changes little, but the time of each iteration is different. Therefore, the comparative experiment fully shows that the acceleration strategy proposed in this paper has high efficiency without loss of accuracy.

## 5. Conclusion

Due to the fact that Magnetic Resonance Imaging (MRI) is currently a very slow imaging technique, its application for dynamic imaging is restricted. The total variation is included into the CS-based MRI reconstruction model, and three regularization requirements are used to ensure that a high-quality reconstructed picture is produced. In this article, a simple yet efficient CS-based optimization model for noisy MRI enhancement is provided. The alternate direction multiplier approach is used to optimize the model, and the *k*-terms power series is applied in order to extract the LogDet function into the augmented Lagrange form. Following this, an approximation of the feature vector is achieved through the iterative process. The quality of the rebuilt picture was substantially better than that of the CS-based MRI image reconstruction method, as shown by experimental results under varied noise settings. The peak signal-to-noise ratio of the reconstructed image was able to be enhanced anywhere from 5 to 20 percent.

## Figures and Tables

**Figure 1:** Schematic diagram of MRI reconstruction. (a) K-space (spectral) image; (b) radial subsampling; (c) MRI image.

**Figure 2:** Comparison of reconstruction performance for different noise. (a) The proposed algorithm; (b) GSCS; (c) NL-CS.

**Figure 3:** Comparison of reconstruction residual for Gaussian noise with *σ*=20. (a) NL-CS, (b) GSCS; (c) the proposed algorithm.

**Figure 4:** Comparison of PSNR of the reconstructed image with the proposed algorithm.

**Figure 5:** Comparison of reconstruction performance for different algorithm. (a) KLLD; (b) SAIST; (c) LSSC; (d) NL-CS; (e) GSCS; (f) the proposed algorithm.

**Table 1:** Reconstruction performance for different noise distribution.

Images		Rayleigh			Gaussian			Nonuniform		
		NL-CS	GSCS	Ours	NL-CS	GSCS	Ours	NL-CS	GSCS	Ours
1	PSNR	31.51	30.23	33.71	35.54	34.29	37.43	29.73	30.11	33.12
	SSIM	0.928	0.934	0.942	0.912	0.920	0.941	0.951	0.955	0.961

2	PSNR	33.11	33.55	33.94	34.06	33.09	33.97	34.53	35.03	35.31
	SSIM	0.889	0.922	0.929	0.825	0.924	0.933	0.9822	0.9125	0.9825

3	PSNR	32.90	33.48	34.02	33.98	33.08	33.91	33.91	34.48	34.74
	SSIM	0.824	0.797	0.763	0.705	0.500	0.561	0.707	0.758	0.825

4	PSNR	30.99	32.42	32.43	32.57	31.55	32.62	33.21	33.82	33.80
	SSIM	0.784	0.815	0.833	0.825	0.817	0.833	0.841	0.8525	0.874

5	PSNR	33.16	34.42	34.97	34.97	33.03	34.93	34.21	31.51	31.85
	SSIM	0.650	0.597	0.663	0.705	0.714	0.561	0.707	0.751	0.821

6	PSNR	37.06	38.11	38.33	38.48	36.61	38.51	35.21	35.11	35.74
	SSIM	0.787	0.815	0.848	0.785	0.819	0.848	0.852	0.8458	0.852

**Table 2:** Reconstruction of average performance for different algorithm.

Average	*σ*	KLLD	SAIST	LSSC	NL-CS	GSCS	The proposed algorithm
SSIM	5	0.914	0.964	0.965	0.923	0.951	**0.966**
	10	0.908	0.934	0.941	0.890	**0.942**	0.941
	20	0.817	0.881	0.883	0.819	0.851	**0.919**
	25	0.815	0.850	0.887	0.793	0.804	**0.892**
	50	0.671	0.713	0.794	0.562	0.572	**0.805**

PSNR	5	36.75	37.30	37.49	37.45	35.89	**37.39**
	10	32.90	33.48	34.02	33.98	33.08	**33.91**
	20	29.01	30.02	30.76	30.69	29.92	**30.77**
	25	27.99	28.88	28.72	29.61	**29.72**	29.71
	50	24.58	25.29	26.46	26.30	26.20	**26.37**

Time/s	10	63.12	30.74	41.75	31.5	75.52	**28.11**

## Data Availability

The datasets used to support the findings of this study are available from the corresponding author upon request.
